# Prognostic Factor Study of Macular Edema Recurrence in Retinal Vein Occlusion after Conbercept Treatment: A Post Hoc Analysis of the FALCON Study

This article has been retracted.

**DOI:** 10.1155/2022/3616044

**Published:** 2022-07-29

**Authors:** Haiying Zhou, Zuhua Sun, Meng Zhao, Xiaoling Liu, Xuan Jiao, Weiwei Zheng, Feng Zhang

**Affiliations:** ^1^Beijing Tongren Eye Center, Beijing Tongren Hospital, Capital Medical University, Beijing Ophthalmology and Visual Sciences Key Laboratory, Beijing 100730, China; ^2^Department of Retina, The Affiliated Eye Hospital, Wenzhou Medical University, Wenzhou, China

## Abstract

**Objective:**

The study was aimed at exploring the potential predictive factors associated with the recurrence of macular edema (ME) secondary to vein occlusion (RVO) after intravitreal antivascular endothelial growth factor (VEGF) loading treatment in the FALCON study.

**Methods:**

This is a post hoc analysis of 30 patients with central RVO and 30 patients with branch RVO. All patients received a monthly administration of intravitreal conbercept during the 3-month loading phase and pro re nata (PRN) treatment during the 6-month follow-up period. Based on the recurrence of ME at the first follow-up visit, patients were classified into the recurrence group or nonrecurrence group. The primary endpoint was to explore the risk factors for recurrence among baseline characteristics, fluorescein angiography (FA) patterns, and optical coherence tomography (OCT).

**Results:**

In general, 38 patients (64.4%) experienced ME recurrence at the first follow-up visit (3 months), regardless of disease type (*p* = 0.32). Significant improvements in VA were noted in both the nonrecurrence and recurrence groups (*p* < 0.001), however, without significant between-group differences (*p* = 0.1). A significant reduction in CRT in both groups (*p* < 0.001) was identified, and patients without recurrence showed a greater reduction in CRT compared with those with recurrence (*p* < 0.001). In addition, logistic regression analyses indicated the corrections of ME recurrence with baseline macular volume and the disruption of the outer limiting membrane at the fovea.

**Conclusion:**

This study suggested that OCT parameters, including baseline macular volume and outer limiting membrane disruption, and reduction in CRT after loading therapy were more predictive of ME recurrence than FA patterns or visual changes following conbercept loading therapy.

## 1. Introduction

Retinal vein occlusion (RVO) obstructs the retinal veins [1] and is the second most common retinal vascular disease after diabetic retinopathy [2]. In general, RVO is commonly divided into central retinal vein occlusion (CRVO) and branch retinal vein occlusion (BRVO) [1]. Thrombosis of the retinal veins increases retinal capillary pressure, capillary permeability, and leakage of fluid and blood into the retina [3, 4]. In patients with RVO, macular edema (ME) is the most common complication and the principal cause of visual impairment [5]. The overproduction of vascular endothelial growth factor (VEGF) is a major cause of the development of ME and hemorrhages [6]. Furthermore, high levels of VEGF promote the progression of retinal nonperfusion and ischemia, which in turn can lead to increased VEGF levels [7], worsening ME and hemorrhages and resulting in subsequent visual impairment. Thus, intravitreal therapy with anti-VEGF is increasingly used to treat ME in patients with RVO [8].

ME is visible on the fundus as increased macular thickness, fluid, or exudates. Fluorescein angiography (FA) can reveal vascular leakage and filling of cystic spaces [9, 10]. However, the gold standard for diagnosing and evaluating ME due to RVO is optical coherence tomography (OCT), a noninvasive imaging tool for macular lesions [11, 12]. Furthermore, central retinal thickness (CRT) is a measure derived from OCT scans and is an essential outcome in clinical trials to assess drug efficacy and vision outcomes [13]. Previous studies have identified the corrections between CRT and visual outcomes after administration of anti-VEGF therapy in patients with ME due to RVO [14, 15].

Conbercept (Lumitin; Chengdu Kang Hong Biotech Co., Ltd., Sichuan, China) is a recombinant fusion protein composed of the extracellular domain 2 of VEGF receptor 1 (VEGFR1) and extracellular domains 3 and 4 of VEGFR2 to the constant region (Fc) of human immunoglobulin G1. This drug binds specifically to various isoforms of VEGF-A, VEGF-B, and placental growth factors [16]. Previous clinical trials noted significant clinical benefits with conbercept in patients suffering from age-related macular degeneration, pathological myopia-associated choroidal neovascularization, or diabetic macular edema (DME) [17–19]. Furthermore, conbercept demonstrated high efficacy and a favorable safety profile in ME secondary to RVO in the phase II FALCON study [20].

Although the efficacy and safety of conbercept were identified previously, there is a lack of investigations on the prognostic factors of ME recurrence after administration of intravitreal anti-VEGF. Thus, we conducted this study to evaluate the association between baseline characteristics, FA patterns, and OCT parameters on ME recurrence after treatment with three consecutive loading doses of conbercept.

## 2. Methods

The data used in this post hoc analysis were obtained during the FALCON study (NCT01809236) [20]. It was a phase II, nonrandomized, noncontrolled, 9-month trial in China to assess the efficacy and safety of intravitreal conbercept in ME secondary to RVO. Patients were recruited from two sites in China, such as the Affiliated Eye Hospital of Wenzhou Medical University and Beijing Tongren Hospital, affiliated to Capital Medical University in China. The study subjects used in this analysis were collected between September 2012 and May 2014. The study complied with the Helsinki Declaration and Good Clinical Practice Guidelines. Each institution's institutional review boards and ethics committee approved the study protocol. All patients provided written informed consent before enrolling in the study.

### 2.1. Participants

The inclusion criteria were as follows: (1) patients were aged 18 years or older; (2) patients had central ME secondary to BRVO or CRVO that had occurred within the past six months; and (3) those had a best-corrected visual acuity (BCVA) of ≤73 Early Treatment Diabetic Retinopathy Study (ETDRS) letters (20/40 Snellen equivalent) and a CRT of ≥320 *μ*m as measured by spectral-domain OCT (Spectralis; Heidelberg Engineering, Heidelberg, Germany). We defined CRVO as an RVO involving four retinal quadrants and BRVO by retinal hemorrhages or other biomicroscopic evidence of RVO and a dilated venous system in two or fewer quadrants of the retina drained by the affected vein. One eye per individual was included in this study.

The exclusion criteria included a relative afferent pupillary defect, prior vitreoretinal surgery, intravitreal anti-VEGF (including but not limited to ranibizumab or bevacizumab) in the study eye within the past six months or in the fellow eye within the past three months, systemic treatment of any anti-VEGF within six months, intraocular or periocular steroid treatment in the study eye within the past three months or systemic steroids within the past one month, reductions in visual acuity from any causes other than RVO, ocular inflammation in either eye, uncontrolled glaucoma (intraocular pressure > 25 mmHg or history of filtration surgery), or treatments using scatter or pan-retinal laser, macular grid laser, or sector laser in the study eye.

### 2.2. Treatment Protocol

A total of 60 patients from the FALCON study in the current research, including 30 ones with BRVO and 30 ones with CRVO. All patients received an administration of intravitreal conbercept (0.5 mg) every month during the loading phase of 3 months. After the loading phase, all patients were followed up monthly for six months. Patients with an increase in CRT by ≥50 *μ*m as compared with the lowest measured value; a loss of ≥5 ETDRS letters compared with the most recent measurement; the presence of new or persistent cystic retinal changes, subretinal fluid (SRF), or neuroepithelial detachment; or the presence of new macular hemorrhage, retinal neovascularization, or any new BRVO received subsequent injections as needed (pro re nata; PRN).

### 2.3. Outcome Measures

The total follow-up time was up to 9 months. Based on the recurrence of ME at the first follow-up visit, all patients were classified into the recurrence group or nonrecurrence group. The primary outcomes were differences between the two groups and risk factors for recurrence among baseline characteristics, FA patterns, and OCT parameters.

We recorded the following data at baseline: (1) demographics; (2) BCVA; (3) intraocular pressure; (4) findings of fundus photography including bleeding and hard exudation in the macular area (Topcon TRC.50-DX; Topcon, Japan); and (5) OCT (HRA-II, Heidelberg, German) including CRT, macular volume (MV), ellipsoid zone (EZ), outer limiting membrane (OLM), disorganization of inner retinal layers (DRIL), SRF, and intraretinal fluid; OCT was measured by mean changes in foveal retinal thickness at all visits (1-9 months) compared with baseline, percentage of subjects with foveal retinal thickness ≤ 250 *μ*m compared with baseline at 3 and 9 months after treatment, and changes in macular edema volume compared with baseline at all visits (months 1-9). (6) Findings of fluorescence angiography (HRA-II, Heidelberg, German) include foveal avascular zone contours, nonperfusion area (NPA), and macular hemorrhage. We assessed BCVA following the ETDRS protocol [21]. Data were collected during the follow-up period using BCVA, FP, and OCT. In order to standardize the reading of Falcon test and ensure the reading quality, each center has carried out cross reading of OCT, FA, and CFP images.

### 2.4. Statistical Analyses

All data were analyzed using R software (version 3.20). Continuous variables are presented as medians with interquartile range (IQR). Person count and percentages describe categorical variables. We compared the baseline ocular characteristics between the two groups, and those characteristics with a *p* value less than 0.3 were included in a binary backward stepwise logistic regression model. We excluded insignificant predictor variables if the Akaike information criterion of the model including this variable was higher when the predictor was not included.

To compare visual acuity and CRT changes between the two groups, we used repeated-measurement analysis of variance and calculated the odds ratio (OR) and its 95% confidence interval (CI). All statistical tests were two-sided. A *p* value of <0.05 was considered statistically significant.

## 3. Results

Among the study subjects, the mean age was 56.7 years, and 33 (55.0%) were male while 30 were diagnosed with CRVO and 30 with BRVO. The median time to onset of disease was 3 months (range, 2–5). Over the 9 months, the total mean number of injections was 7.59 ± 1.39 for CRVO and 7.14 ± 1.90 for BRVO.

At baseline, as compared with patients with BRVO, patients with CRVO showed significantly poorer vision (BCVA [ETDRS letters], 48.73 ± 15.9 in CRVO vs. 57.83 ± 13.42 in BRVO, *p* = 0.02), a higher CRT (695.5 *μ*m [IQR, 592-916] in CRVO vs. 549.5 *μ*m [IQR, 467-656] in BRVO, *p* = 0.0002), a larger MV (13.79 mm^3^ [IQR, 11.81-17.41] in CRVO vs. 12.35 mm^3^ [IQR, 11.27-13.85] in BRVO, *p* = 0.015), a smaller area of macular NPA (*p* = 0.0007), a lowerr proportion of macular hemorrhage (66.7% vs. 96.7%, *p* = 0.006), and a higher proportion of cystoid macular edema (CME; 96.7% vs. 53.3%; Table 1).

One patient with CRVO was lost to follow-up one month after the loading phase and was, therefore, not included in the subsequent analysis. When we compared the baseline BCVA to that at the first follow-up visit, we considered a gain of ≥15 ETDRS letters from baseline as an improvement, <15 letters as vision maintenance, and a loss of ≥15 ETDRS letters as a worsening disease. Among the patients with CRVO, 12 eyes (41.38%) showed improvement, 16 (55.17%) eyes showed no change, and 1 (3.35%) eye worsened. Among those with BRVO, 17 (56.67%) eyes improved, 13 (43.33%) eyes showed no change, and no eyes worsened. No statistically significant differences were found between the two groups in vision changes. After the loading phase, changes in CRT from baseline were greater for patients with CRVO than for those with BRVO (−339.0 *μ*m [IQR, 219.0] vs. −274.5 *μ*m [IQR, 198.0], *p* < 0.001). The vision changes between male and female were without statistical difference (14.0 letters [IQR, 8.0] vs. 10.5 letters [IQR, 12.3], *p* = 0.10). Neither was found in CRT changes (−307.0 *μ*m [IQR, 259.0] vs. −298.5 *μ*m [IQR, 142.0], *p* = 0.34).

After the loading phase, 38 patients (63.3%) experienced ME recurrence and required redosing at the first visit after the loading phase. Among these, 17 patients (56.7%) had BRVO and 21 (70%) had CRVO, and the recurrence was independent of disease type (*p* = 0.32). Among the patients who received redosing, the BCVA at baseline, last examination during the loading phase, and first follow-up visit were 57 letters (IQR, 11), 72 letters (IQR, 12), and 74 letters (IQR, 13), respectively. For those who had not yet needed additional injections, the BCVA at baseline, last examination during the loading phase, and first follow-up visit were 59 letters (IQR, 25), 69 letters (IQR, 27), and 71.5 letters (IQR, 27.8), respectively. However, there were significant improvements in vision in both groups (*p* < 0.001) and no significant differences among groups (Figure 1(a)). Similarly, CRT was significantly lower in both groups (*p* < 0.001; Figure 1(b)). However, patients who did not experience recurrence had a greater CRT reduction than those who received redosing (*p* < 0.001; Figure 2). Among the patients with a recurrence of ME, the CRT at baseline, last examination during the loading phase, and first follow-up visit were 634.5 *μ*m (IQR, 206.2), 329 *μ*m (IQR, 231.5), and 288.5 *μ*m (IQR, 142), respectively. For those who did not yet require additional injections, the CRT at baseline, last examination during the loading phase, and first follow-up visit were 573.0 *μ*m (IQR, 195.0), 245 *μ*m (IQR, 29), and 244 *μ*m (IQR, 28), respectively.

In this study, the baseline MV significantly correlated with the recurrence of ME at the first visit after the loading phase (OR = 1.44, 95% CI, 1.08–1.92; *p* = 0.01; Table 2). In addition, a significant correlation between the presence of disrupted OLM at the fovea and recurrence of ME was identified (OR = 0.17, 95% CI 0.05–0.64; *p* = 0.008). We detected no significant association between ME recurrence and FA patterns, including irregular FAZ contours, NPA, or macular hemorrhage (Table 2). Patients who required redosing showed a trend toward a higher baseline CRT as compared with patients who did not yet require additional doses (634.5 *μ*m [IQR, 207] vs. 573.0 *μ*m [IQR, 195]; *p* = 0.07, Table 2). Because the CRT and MV can be confounding variables and because we established a linear correlation between CRT and MV in this study (*p* < 0.001, *R*^2^ = 0.75), we used the baseline MV instead of the CRT as the independent variable in the multinomial regression analyses to determine the correlations with ME recurrence. These factors were subjected to logistic regression analysis. In this model, the Akaike information criterion was 68.5, and the area under the curve was 0.789 (Figure 3).

## 4. Discussion

Previous studies demonstrated the efficacy and safety of intravitreal injection of conbercept to treat ME secondary to RVO. Such clinical benefits consistently improved visual acuity and anatomic endpoints in both BRVO and CRVO groups. In the FALCON study, these improvements persisted and even improved with PRN dosing during the follow-up period [20]. However, in that study, the response to conbercept treatment varied among individuals in patients with ME secondary to RVO. After the loading phase, ME persisted in some eyes, and subsequent injections were required. Among the patients who experienced a ME resolution, some experienced ME recurrence and required repeated injections. Because the prediction of ME recurrence is clinically essential for long-term outcomes in patients with ME secondary to RVO, this post hoc study to identify predictive factors associated with ME recurrence was conducted. Baseline characteristics and related data at the first follow-up visit from the FALCON study were collected and analyzed. Considering that a similar proportion of patients with BRVO and CRVO received PRN dosing after the loading phase, we included patients with both BRVO and CRVO in this study.

OCT is one of the most common imaging modalities for assessing the efficacy of therapeutics in ME secondary to RVO [22]. The CRUISE and BRAVO studies reported a rapid reduction in CRT within one week after ranibizumab treatment. The mean CRT reduction from baseline to 6 months was −435 *μ*m (0.3 mg) and−453 *μ*m (0.5 mg) in CRVO patients and −339 *μ*m (0.3 mg) and −345 *μ*m (0.5 mg) in BRVO patients, respectively [23, 24]. In the BRAVO study, OCT images at month 3 of ranibizumab treatment provided predictive information for patients with CRVO but not for those with BRVO [25]. In particular, poorer vision outcomes at 6 and 12 months were associated with persistent CME and a central foveal thickness of ≥250 *μ*m at 3 months. Our study found a significant reduction in CRT and an improvement in VA in both groups after the loading phase. At the first follow-up visit, changes in CRT from baseline were −339.0 *μ*m in CRVO patients and −274.5 *μ*m in BRVO patients. Concomitantly, a VA gain of ≥15 ETDRS letters was achieved in 41.38% of patients with CRVO and in 56.67% of patients with BRVO.

Several studies have investigated the OCT parameters related to ME recurrence. For example, in eyes with BRVO, cystic macular changes and DRIL with ME recurrence were identified [26–28]. Although the baseline CRT was not significantly related to ME recurrence (*p* = 0.07) in our study, patients without recurrence had a greater reduction in CRT than those with recurrence after loading therapy (*p* < 0.001). Moreover, logistic regression analysis showed that the baseline MV significantly correlated with ME recurrence at the first visit after the loading phase. Because MV is a more comprehensive ME indicator than CRT especially for the perifoveal regions, MV can be adopted as a prognostic factor for ME secondary to RVO. In addition, because we established a linear correlation between CRT and MV in this study, CRT could be a confounding variable to MV in ME prognosis. Notably, for subanalysis, no significant differences were identified between genders.

In addition to measuring the central foveal thickening of the macula edema, the OCT system allows the microretinal structures to be visualized, including the OLM and EZ. In particular, previous studies identified the correction of disruption in the OLM with poor visual prognosis after RVO treatment [29–32]. However, in a recent study that collected and analyzed the data of 381/301 BRVO/CRVO naive patients from the BRIGHTER and CRYSTAL studies, only CRT and age were associated with visual prognosis instead of OLM disruption or DRIL [15]. In our study, we noted a significant correlation between baseline OLM disruption at the fovea and ME recurrence, suggesting that baseline OLM integrity could serve as a predictor for recurrence of ME. The OLM is a linear confluence of junctional complexes between Muller cells and photoreceptors [33]. In addition, the OLM separates the layers of rods and cones from the overlying outer nuclear layer and serves as a barrier against macromolecules [34]. A prior study demonstrated the presence of tight junctions (TJs) in the OLM and between the glial Muller cells and photoreceptors in rat and monkey retinas [35]. Occludin, an integral membrane protein that localizes at the TJ [36], was organized between the glial Muller cells and the photoreceptors. Occludin expression decreased, and glial Muller cells swelled in DME at the OLM level [37]. These findings suggest that the OLM could be a part of the retinal barrier, and its disruption could result in fluid retention and consequent edema. Although anti-VEGF treatment can restore the barrier effect of the OLM [38, 39], recurrent episodes of edema occur when baseline damage to the OLM is too severe to be restored.

Clinically, FA remains an essential tool for detecting morphologic changes in the retinal vasculature and provides a functional evaluation of the extent of macular ischemia, vascular leakage, and neovascularization [11]. As reported by the SCORE study, in patients with BRVO, nonperfusion was the only significant baseline factor for neovascularization [40].

The WAVE study revealed a relationship between retinal ischemia and ME severity, as reflected by central macular thickness [41]. In addition, the correlation between FA patterns and ME recurrence was also investigated. According to a previous study, the central NPA and parafoveal NPA of the superficial capillary plexus strongly correlated with ME recurrence in BRVO patients who received intravitreal anti-VEGF treatment [42]. Similarly, BRVO patients with NPA of more than half of the 1 mm zone of the ETDRS should be monitored closely for ME recurrence within six months of intravitreal bevacizumab injection [43]. Furthermore, patients with BRVO who have significant nonperfusion may require repeated dosing of dexamethasone [44]. Given these, we investigated the relationship between baseline FA patterns and the early recurrence of ME after loading treatment with conbercept. Interestingly, neither the NPA nor macular hemorrhage was associated with ME recurrence at the first follow-up visit. Although this preliminary finding did not support the predictive value of FA in the early recurrence of ME, a longer follow-up period and a larger sample size are required to further evaluate its prognostic value in VA outcomes.

However, this study has several inherent limitations, such as a small cohort size, a lack of long-term data to rule out the possibility of MV remission after four injections, and a lack of systemic collection of baseline characteristics. All of these factors may result in biases and affect the power and significance of the findings. In the future, long-term prospective cohort studies should be conducted to validate the findings and may obtain more study insights.

This study suggests that OCT parameters are more predictive of ME recurrence than FA patterns or visual changes after conbercept loading therapy. Significantly, baseline MV, OLM disruption, and reduction in CRT after anti-VEGF loading therapy could be valuable tools in clinical practice for predicting future recurrence in patients with RVO-related ME.

## Figures and Tables

**Figure 1:** Clinical changes of visual acuity and central retinal thickness in recurrent and nonrecurrent patients after the loading phase. (a) The BCVA (ETDRS letters) at baseline, 3 month (last examination during the loading phase), and 4 months (first follow-up visit). (b) The CRT at baseline, 3 months, and 4 months. Median value was presented with IQR for error bars.

**Figure 2:** Patients without recurrence showed a greater reduction of CRT compared to those with recurrent ME and treatment of redosing. The CRT was measured for patients in both groups at baseline, 3 months (last examination during the loading phase), and 4 months (first follow-up visit). Median value was presented with IQR for error bars.

**Figure 3:** Receiver operating characteristic curve of logistic regression analysis. Baseline macular volume and OLM disruption were identified as predictive factors.

**Table 1:** Baseline characteristics of the study subjects.

Features	CRVO (*n* = 30)	BRVO (*n* = 30)	*p* value
Mean BCVA (ETDRS letters)	48.73 ± 15.91	57.83 ± 13.42	0.02
CRT (median, IQR)	695.5 (592–916)	549.5 (467–656)	0.0002
MV (median, IQR)	13.79 (11.81–17.41)	12.35 (11.27–13.85)	0.015
Regular FAZ contours^1^, *n* (%)	15 (50.0%)	8 (26.7%)	0.07
Nonperfusion area (NPA)^2^			0.0007
No NP, *n* (%)	13 (43.33%)	1 (3.33%)	
<5 PD, *n* (%)	5 (16.67%)	8 (26.67%)	
>5 PD, *n* (%)	9 (30.00%)	17 (56.67%)	
Macular hemorrhage, *n* (%)	20 (66.67%)	29 (96.67%)	0.006
Macular HE, *n* (%)	3 (10.00%)	7 (23.33%)	0.3
EZ			0.76
Intact, *n* (%)	5 (16.67%)	8 (26.67%)	
Disruption in the fovea, *n* (%)	13 (43.33%)	15 (50.00%)	
Disruption in the parafovea, *n* (%)	2 (6.67%)	4 (13.33%)	
Unevaluable, *n* (%)	10 (33.33%)	3 (10.00%)	
OLM		(0.00%)	0.86
Intact, *n* (%)	8 (26.67%)	8 (26.67%)	
Disruption in the fovea, *n* (%)	10 (33.33%)	14 (46.67%)	
Disruption in the parafovea, *n* (%)	3 (10.00%)	5 (16.67%)	
Unevaluable, *n* (%)	9 (30.00%)	3 (10.00%)	
DRIL^3^, *n* (%)	10 (33.33%)	11 (36.67%)	0.99
IRF			0.0004
No IRF, *n* (%)	0 (0.00%)	1 (3.33%)	
Macula area, *n* (%)	1 (3.33%)	10 (33.33%)	
Paramacular area, *n* (%)	0 (0.00%)	3 (10.00%)	
CME, *n* (%)	29 (96.67%)	16 (53.33%)	
SRF			0.73
No SRF, *n* (%)	10 (33.33%)	8 (26.67%)	
Small amount, *n* (%)	16 (53.33%)	16 (53.33%)	
Large amount, *n* (%)	4 (13.33%)	6 (20.00%)	

^1^Two unevaluable patients were not included in the analysis. ^2^Six patients with bleeding events were not included. ^3^Six patients with unevaluable DRIL were not included. SD: standard deviation; IQR: interquartile range; BCVA: best-corrected visual acuity; CRT: central retina thickness; MV: macular volume; FAZ: foveal avascular zone; NPA: nonperfusion area; PD: papilla diameter; HE: hard exudates; EZ: ellipsoid zone; OLM: outer limiting membrane; DRIL: disorganization of retinal inner layers; IRF: intraretinal fluid; CME: cystoid macular edema; SRF: subretinal Fluid.

**Table 2:** Clinical measurements comparisons of the study eyes between the recurrence group and nonrecurrence group.

Features	Recurrence group (*n* = 38)	Nonrecurrence group (*n* = 21)	*p* value
Disease type			
BRVO, *n* (%)	17 (44.74%)	13 (61.90%)	0.32
CRVO, *n* (%)	21 (55.26%)	8 (38.10%)	
BCVA (ETDRS letters), median (IQR)	59 (25)	57 (11)	0.32
CRT, median (IQR)	634.5 (207)	573.0 (195)	0.07
MV, median (IQR)	13.04 (4.41)	11.41 (3.25)	0.01
Irregular FAZ contours, *n* (%)	24 (63.16%)	11 (52.38%)	0.75
NP			
No NP, *n* (%)	10 (26.32%)	4 (19.05%)	0.003
<5 PD, *n* (%)	7 (18.42%)	6 (28.57%)	0.18
>5 PD, *n* (%)	16 (42.11%)	10 (47.62%)	0.003
Unevaluable, *n* (%)	5 (13.16%)	1 (4.76%)	0.47
Macular hemorrhage, *n* (%)	8 (21.05%)	2 (9.52%)	0.47
EZ			
Intact, *n* (%)	8 (21.05%)	5 (23.81%)	0.099
Disruption in the fovea, *n* (%)	14 (36.84%)	14 (66.67%)	0.03
Disruption in the parafovea, *n* (%)	5 (13.16%)	1 (4.76%)	0.41
Unevaluable, *n* (%)	11 (28.95%)	1 (4.76%)	0.04
DRIL			
No, *n* (%)	19 (50.00%)	14 (66.67%)	0.27
Yes, *n* (%)	15 (39.47%)	5 (23.81%)	<0.001
Unevaluable, *n* (%)	4 (10.53%)	2 (9.52%)	0.99
OLM			
Intact, *n* (%)	10 (26.32%)	6 (28.57%)	0.99
Disruption in the fovea, *n* (%)	11 (28.95%)	13 (61.90%)	0.02
Disruption in the parafovea, *n* (%)	7 (18.42%)	1 (4.76%)	0.23
Unevaluable, *n* (%)	10 (26.32%)	1 (4.76%)	0.08
IRF			
No IRF, *n* (%)	0 (0%)	1 (4.76%)	0.36
Macula area, *n* (%)	5 (13.16%)	6 (28.57%)	0.17
Paramacular area, *n* (%)	2 (5.26%)	1 (4.76%)	0.99
CME, *n* (%)	31 (81.58%)	13 (61.90%)	0.12
SRF			
No SRF, *n* (%)	11 (28.95%)	7 (33.33%)	0.77
Small amount, *n* (%)	21 (55.26%)	11 (52.38%)	0.99
Large amount, *n* (%)	6 (15.79%)	3 (14.29%)	0.99

IQR: interquartile range; BCVA: best-corrected visual acuity; CRT: central retina thickness; MV: macular volume; FAZ: foveal avascular zone; NPA: nonperfusion area; PD: papilla diameter; HE: hard exudates; EZ: ellipsoid zone; OLM: outer limiting membrane; DRIL: disorganization of retinal inner layers; IRF: intraretinal fluid; CME: cystoid macular edema; SRF: subretinal fluid.

## Data Availability

All the raw data used to support this study are available by contacting the corresponding author upon request.
